# Impact of Mo^+2^ addition and thermal annealing on the surface morphology, electrical transport properties and Mott's parameters of WO_3_ films for potential photonic devices

This article has been retracted.

**DOI:** 10.1016/j.heliyon.2024.e36783

**Published:** 2024-08-23

**Authors:** S.M. Alshomar, Mohamed S. Attia, Alaa Ahmed Akl, Naglaa Fathy, Hissah Saedoon Albaqawi, Hira Affan, Ehab Sabry Mohamed, Lamiaa G. Amin, Safwat A. Mahmoud

**Affiliations:** a Department of Physics, College of Science, University of Hail, Box 2440, Hail, Saudi Arabia; b Chemistry Department, Faculty of Science, Ain Shams University, Abbassia, Cairo, 11566, Egypt; c Physics Department, Faculty of Science, Minia University, Minia, 111559, Egypt; d Physics Department, Faculty of Science and Humanities, Ad-Dawadmi, Shaqra University, Saudi Arabia; e Department of General Courses, College of Humanities and Social Sciences, Northern Border University, Arar, 91431, Saudi Arabia; f Department of Combat and Individual Sports, Faculty of Physical Education, Tanta University, Tanta, Egypt; g Physics Department, Faculty of Science, Northern Border University, Arar, 13211, Saudi Arabia

**Keywords:** Conductivity mechanisms, Mott's parameters, Thin solid films, Metal transition oxides

## Abstract

This work investigates the compositional dependence and thermal annealing of the morphological properties, electrical conductivity mechanisms and Mott's parameters of sprayed Mo_x_W_1-x_O_3_ (x = 0, 0.05, 0.10 and 0,20) thin films. The prepared thin films were examined using field emission scanning electron microscopy (FE-SEM), energy dispersive X-ray analysis (EDX) and Fourier transform infrared spectroscopy (FTIR) techniques. In addition, the two-point probe method was used to calculate the electrical properties of Mo_x_W_1-x_O_3_ thin films. The FTIR results revealed that; the tungsten hydroxyl bond (W-OH) and the surface hydroxyl group vibrated within the ranges of 1558.62–1645.56 cm^−1^ and, 3296.76 and 3424.34 cm^−1^, respectively. Furthermore, a prominent band in the spectrum spanning from 850 to 650 cm^−1^ represents the W-O-W bridge mode. The FE-SEM investigations found that the molybdenum (Mo) dopant caused significant changes in the surface morphology of the films. The EDX results showed that the percentages of the isotropic elements Mo_x_W_1-x_O_3_ agreed well with those obtained by atomic weight. Studies of the conduction mechanism indicate that the transition temperature was approximately 393K. Corresponding to Mott's model, the conduction mechanism below this temperature was across the variable hopping conduction band near the Fermi level. The mechanism exhibited a cycle of localised states through activated thermionic emission above 393K. Mott parameters were also estimated in addition to barrier potential energies, trapping state energies, local state densities, and other variables. The results revealed that both temperature areas had a rise in ρ_o_ and ρ_1_ values during and after annealing. The ΔE_o_ and ΔE_1_ values in each temperature area decreased as the Mo-ion concentration increased. Furthermore, the conversion temperature gradually reduced as Mo was added. Based on these properties, the study's overall findings indicate that Mo_x_W_1-x_O_3_ is suitable for future photonic devices and optoelectronic applications.

## 1 Introduction

In amorphous, poly-, micro-, and nanocrystalline semiconductor materials, the control of direct electrical characteristics is contingent upon the effective trapping of influence at defects situated inside the bulk of the layer. Regarding the spatial distribution of structural defects, several studies have investigated carrier transport in thin film layers that have a high defect density and are almost uniformly distributed. The development of functional materials that are capable of generating electrical energy from diverse sources, including solar, wind, hydropower, biomass, and thermal energy, represents a central focus of contemporary research endeavours [1,2]. However a substantial quantity of waste heat is inevitably produced within the surrounding environment by leveraging these varied technologies to generate electricity. Consequently, numerous researchers have directed their efforts towards the direct conversion of thermal energy into electrical energy, and vice versa when employing thermal energy to produce electrical power [3]. Meanwhile, applications for thermoelectric materials span a broad spectrum, encompassing power generation, temperature sensing, electronic device cooling, and infrared cooling sensor technologies. Furthermore, thermoelectric materials are extensively utilised in devices designed to convert thermal energy directly into electricity [4].

The most relevant transport mechanism describing the electrical properties of amorphous, micro- or nano-crystalline semiconductors is carrier waves switching between local states near the conduction band edge (E_C_) a mechanism first suggested by Mott [5,6]. Large monocrystalline grains that have a columnar structure make up polycrystalline layers (100 nm and thicker), and it is generally acknowledged that flaws are primarily found grain borders. Thus, in this case, the intergranular barriers resulting from the carrier trapping effect at these grain boundaries have a significant impact on carrier transit, in accordance with to Seto's theory [[7], [8], [9], [10]]. Bulk defects usually result from two main causes, namely, strained bonds and dangling bonds that correspond to the bandgap's shallow and deep level trap states. Gaussian distribution with the maximum at the middle gap is the most significant distribution type that characterises this situation and the residuals' exponential band tailing for type defects, mainly corresponding to strained and dangling bonds, respectively. Several methods have also been proposed to determine these distributions based on conduction activation energy, resistivity, low-frequency noise and capacitance measurement.

The associated energy distribution of the states (DOS) dictates the material's crystal quality and production parameters; thus, numerous studies have attempted to identify the DOS as a diagnostic tool [11,12].

Mo^+2^ has a +2 charge, whilste W -in WO_3_ has a +6 charge. When Mo^+2^ substitutes for W in the WO_3_ crystal lattice, it creates electron deficiencies that act like positive charges and help improve the electrical conductivity in WO_3_. This can be beneficial for applications such as photocatalysis or gas sensing. Doping with Mo^+2^ can also alter the bandgap of WO_3_. In particular, the bandgap might be narrowed by introducing Mo^+2^. This can be useful for applications such as photoelectrochemical cells, where a narrower bandgap allows WO_3_ to absorb a wider range of light for efficient light-to-electricity conversion. Mo itself is a good catalyst for various reactions. Doping WO_3_ with Mo^+2^ can introduce catalytic sites and improve its overall catalytic activity. This could be beneficial for applications, including the degradation of pollutants or hydrogen production. Furthermore, in terms of ionic size, Mo^+2^ has a similar ionic radius to W^+6^, allowing for good integration of molybdenum (Mo) into the WO_3_ lattice without causing significant strain or defects. This is important for maintaining the overall structure and functionality of WO_3_ [13,14].

Notably, the specific reasons for choosing Mo^+2^ doping can vary depending on the desired application and the specific properties that researchers want to achieve.

Mo_x_W_1-x_O has a broad range of potential technological applications in many photovoltaic devices, such as optical switching coatings, displays and smart windows [15]. Similarly, WO_3_ has numerous promising photocatalytic applications [15], and can be used in gas chromic devices [16], water splitting [15,17], memory devices [15,18], photochromic devices [19], and biomedical applications [20], among others. With these applications, it is critical to understand that the processing parameters, content, and shape of Mo_x_W_1-x_O thin films all have an impact on their respective applications. Current research focuses on new and intriguing applications of these versatile materials.

A central focus of contemporary research efforts is on comprehensively comparing the preparation methods and properties of wide-bandgap oxide thin films with those of alternative material types. Some studies have also investigated the electrical conductivity of wide-bandgap materials and the impact of thermal annealing on this critical physical parameter across varying compositions. Concurrently, the pursuit of high-performance thermoelectric materials with a broad range of bandgap energies has been extensively explored and investigated by the scientific community.

Amongst the more recently developed thermoelectric materials utilised in thermal applications are Be-Te based alloys. At temperatures of up to 450 K, the primary applications for n-type and p-type thermoelectric systems lie within the realms of waste heat recovery and cooling [21,22]. Conversely, lead-based alloys are more suitable for the intermediate temperature range of 500–900 K [23]. For applications that require operational temperatures exceeding 900 K, thermal generators comprising silicon and germanium alloys are commonly employed. However, despite the continued high demand for Be-Te and, Pb-Te based alloys, as well as silicon-germanium alloys as materials for commercial thermal power generators and refrigeration systems, the environmental concerns associated with the hazardous nature of bismuth and lead-based alloys have hindered their widespread adoption across numerous applications. As a complement to the current study, the effect of increasing the amount of Mo-ion on microstructural properties, crystal defects, optical preparations and refractive index scattering parameters of thin films of Mo_x_W_1-x_O_3_ (0 % ≥ x ≥ 20 %) were examined by the authors in a previously published paper [11,12,24].

Carrier concentration and carrier mobility are two critical parameters that have a significant impact on semiconductor electrical conductivity. For Mo_x_W_1-x_O_3_, doping with Mo^+2^ acts as a beneficial impurity in WO_3_. Mo atoms have one more valence electron than tungsten atoms. When incorporated into the WO_3_ lattice, this extra electron becomes a free carrier, increasing the overall carrier concentration and making the material more conductive. The effect of Mo on mobility can be somewhat complex. In some cases, it can introduce defect scattering sites and reduce mobility. However, optimised doping levels, Mo can also help improve the crystal structure and enhance mobility. In general, by carefully controlling the amount of doped Mo^+2^ doped, a significant increase in the electrical conductivity of WO_3_ can be achieved for various applications.

Therefore, this study aimed to investigate the influence of thermal annealing and Mo-ion amount in WO_3_ films on the activation energies, the mechanism of Mott's parameters and electrical conductivity, such as density of the localised states at the phonon frequency, Fermi level, residual electrical conductivity, characteristic temperature, average hopping distance, and hopping energy. The potential conduction mechanisms were investigated, estimate Mott's parameters, potential barrier energies, the density of the localised states, trapping state energies and other relevant characteristics were estimated. The authors also aimed to identify pre-exponential factors (ρ_o_ and ρ1) and their associated activation energies. Notably, the authors faced difficulties collecting comparable data for comparing our results with those of the other works due to the lack of such as in earlier studies pertaining to the analysis of Mo_x_W_1-x_O_3_ films.

## 2 Experimental details

### 2.1 Preparation of W_1-x_Mo_x_O_3_ thin films

Appropriate preparation conditions were selected in the system to produce a single tungsten oxide phase (WO_3_) thin films using a chemical spray pyrolysis technique. High quality thin films must have pinhole-free surface morphologies, good roughness and strong adhesion to the glass substrate's surface. Mainly, ammonium paratungstate [((NH_4_)_10_(W_12_O_41_)·5H_2_O)] (99 %, Sigma Aldrich), and ammonium metamolybdate [(NH_4_)_6_Mo_7_O_24_] (98 %, Thomas Baker) were combined with 100 mL of hot distilled water at 333K to create the initial aqueous chemical solution, which had a concentration of 0.01 mol.

Ammonium metamolybdate was used to add Mo ions to pure tungsten trioxide to achieve Mo ion doping in WO_3_ at 0 %, 2 %, 5 %, 10 %, and 20 %. Ammonium paratungstate and ammonium metamolybdate were dissolved in 100 mL of distilled water to create the chemical solution, which was after that used to create the doped thin films. Next, the doped thin films were annealed for 2 h at 823K in a vacuum [11,12,24].

Apart from using a nozzle's with a diameter of 0.7 mm, the preparation conditions during the thin film deposition included a distance of 40 cm between the film and the substrate, a flow rate of 4 mL/min, and a concentration of 0.01 M for the solution. The film thickness was fixed at 650 nm, and the deposition time for all samples was set at 10 min. The glass substrates were washed and cleaned in methanol solution using an ultrasonic cleaner for 5 min before being dried with hot air. The films were created on glass substrates preheated at 673K. The thin films were calibrated, and the film thickness was calculated by means of a simple mechanical technique using a sharp stylus on the border of the deposited part of the film.

### 2.2 Electrical resistivity measurement

Measuring the electrical resistivity of thin films is crucial for characterising their electrical behaviour. The following is a breakdown of the systems and the potential errors involved: First, the four-probe method, which is the most common technique, uses four electrical contacts on the film to separate current flow from voltage measurement, thus eliminating contact resistance errors. A constant current is applied through two outer probes, and the voltage drop is measured between the two inner probes. Second, the Van der Pauw method uses four ohmic contacts placed in a specific pattern (often cloverleaf-shaped) on a thin film with uniform thickness. Doing so facilitates resistivity measurement, regardless of the sample shape, and eliminates errors due to non-uniform current distribution.

At the same time, there are possible errors in these previous methods, For instance, i- Imperfect connections between the probes and the film can introduce additional resistance, which affects affecting the measured value. Current leakage through the substrate or surrounding environment can lead to underestimation of the film's resistivity, whilst variations in film thickness can cause inaccurate resistivity calculations. Techniques such as profilometry can help measure thickness accurately. However, the resistivity of most materials changes with temperature. Furthermore, it is important to maintain controlled temperature environment during measurement. By understanding these factors and choosing the appropriate measurement system, accurate and reliable data on the electrical resistance of thin films can be obtained [[25], [26], [27], [28]].

Using a two-point probe method, the electrical resistance of the suitable Mo_x_W_1-x_O_3_ thin films was measured. A specially designed metal sample holder was used to measure DC resistance as two aluminum electrodes were deposited on the uncoated portions of the Mo_x_W_1-x_O_3_/glass samples in the middle of the film. To improve the contact between the load spring and the two aluminum poles, it was fastened onto two copper rods. Using a digital Keithley scale (model 616) and a stable power source, the electrical impedance of the samples was measured. A K-type thermocouple made of "chromel alumel" alloys in close thermal contact with a sample surface was also used to measure the sample temperature. The temperature was measured and recorded, and its dependence on the continuous electric current passing through the samples was also identified. The specific electrical resistivity, ρ_dc_ of the studied thin films were in the temperature range of 293–523 K. These values were calculated experimentally using Eq. (1).

(1) $$\rho_{DC}=\frac{R.w}{d}.t$$

where R is the resistance of the thin film (Ω), w is the length of the film covered electrode (the thin film width is 2.5 cm), t is the thickness of the thin film (cm) The cross-sectional area of thin films is equal to the product of w multiplied by t in centimeteres and d is the separation distance between the two copper electrodes which represents length (1.4 cm).

### 2.3 FTIR spectroscopy

Using a Diamond Crystal ATR (attenuated total internal reflection) accessory, a Bruker Alpha II FTIR spectrometer was used to examine samples with 0 %, 5 %, 10 %, and 20 % Mo concentrations. Direct measurements of liquid and solid samples can be performed without using specialised samples or a salt plate. In addition, Opus 7.8 software was installed to operate the spectrometer.

### 2.4 FE-SEM and EDX

The morphological characteristics of the Mo_x_W_1-x_O_3_ thin-film were investigated using a Zeiss SIGMA VP field emission scanning electron microscope (FE-SEM) manufactured in Germany. The present samples' compositional elements were examined using standard ZAF corrections. Furthermore, an X-ray spectroscope (Oxford Instruments, England) coupled with a Zeiss–SIGMA VP microscope (Germany) was used to analyse the examined samples using energy-dispersive X-ray spectroscopy.

## 3 Results and discussion

### 3.1 FE-SEM and EDX analysis of Mo_x_W_1-x_O_3_ thin films

The recent years have seen a huge increase in the use of the FE-SEM technology, which is typically employed to examine the morphological and structural properties of materials, especially those that are at the nanoscale. When evaluating material morphology, many researchers prefer FE-SEM over scanning electron microscopy (SEM), as the former produces a clearer image with increased magnification and resolution, thus revealing every detail. Furthermore, the surface characteristics of the examined samples can be successfully scanned and analysed, regardless of whether they are crystalline, granular, smooth, or rough [[29], [30], [31]]. In addition, describing the FE-SEM images provides useful information regarding the surface of the sample under study. FE-SEM can produce high-resolution images when operated at low accelerating voltages; in fact, it is better to use lower acceleration voltages, as they are more suitable for the microscopic analysis of sensitive materials. In addition, a sample with regular and homogenous crystalline sizes or grains typically has a smooth surface. A material with a smooth and homogeneous surface exhibits high conductivity, low absorption and high transmittance along with low reflection. In Comparison, a sample with a rough and heterogeneous surface usually has physical properties below the required threshold, has low transmittance and conductivity, and has a high ability to absorb and reflect light. These defects should be avoided [29,30].

In terms of the effect of the addition of Mo-ions on the surface morphology of the samples made from WO_3_, the results showed that the surface morphology of the pure WO_3_ film's surface morphology, as shown in Figure 1A, had an island-like composition made up of teeny fine grains. When 20 % Mo is added, the film's morphology changes to a dense network of islands with roots that resemble nests. Consequently, the 20 % Mo-doped film's enhanced cross-linked channels provide broad paths for ions to readily spread into the film lattice, as well as accelerated kinetics that enhanced the films' electrical performance [32].

**Fig. 1:** *The FE-SEM images and the composition elemental (EDX) patterns of (A) Mo (0 %) dop*ed WO3 and (B) Mo (20 %*) doped WO*_*3*_.

One effective method for examining the components of chemical compounds is through energy dispersive X-ray spectroscopy (EDX), particularly when examining the ratios of the weaker elements. This is accomplished by measuring the intensity of the X-rays emitted by those elements because of their excitation from exposure to the energy of the electron beam. To read the weaker and less intense X-rays produced, highly sensitive meters must be present. The proportion of the components of the elements present in the sample is determined by comparing it to the recorded standard data. This dataset also includes a database containing all the wavelengths of all elements, beginning with an atomic weight equal to 3. As demonstrated in Fig. 1B, the EDX spectra of a sample that was both undoped and doped with 20 % Mo were measured to ascertain the percentage of the three element components that were uniformly distributed, namely, Mo, W, and O. These measurements also unmistakably show the existence of Mo in the WO_3_ host lattice. In addition, the samples were analysed at room temperature by electron microscopy in different regions of the sample, after which the average values were considered. EDX analysis was implemented to allocate the samples' overall compositional constituents to specific areas of the sample surface.

Clearly, there is a good match between the proportion of discovered components (Mo, W, and O) and those selected through experimentation. This finding is completely corroborated by the results, listed in Table 1, which indicate that the 20 % Mo sample and the uncoated sample are single-phase samples free of other elemental impurities. It is also evident that the percentages of oxygen are slightly higher than the atomic ratios. When a sample is cooled to room temperature, a small amount of oxygen may be taken up from the surrounding air, which could explain the slight excess oxygen in the sample [33]. The results also reveal a similar behavior, in which the oxygen stoichiometric measurement is generated, in accordance with what has previously been reported for comparable samples [34]. With an accuracy of roughly 0.1 %, compositional element analysis with an EDX spectrometer generally yields a good assessment of the sample under examination. Overall, there is strong agreement between the theoretically calculated and experimentally obtained proportions.

**Table 1:** The compositional elements percentages determined by EDS technique**.**

*Mo*_*x*_*W*_*1-x*_*O*_*3*_	*Weight%*				*Atomic%*			
	*Mo*	*W*	*O*	*Total*	*Mo*	*W*	*O*	*Total*
X = 0.00	0.00	79.10 ± 2.5	20.90 ± 2.3	100	0.00	79.30 ± 3	20.70 ± 2.2	100
X = 0.20	9.63 ± 2.8	72.78 ± 2.5	17.59 ± 2.3	100	8.96 ± 2.8	64.64 ± 3	22.40 ± 2.2	100

### 3.2 FTIR analysis of Mo_x_W_1-x_O_3_ thin films

FTIR is a kind of analytical method used to examine the characteristics of molecules in a sample material. FTIR spectroscopy offers useful insights into the chemical structures of nanomaterials and presents its results though an ‘infrared spectrogram’, graph that displays the amount of light absorbed by a material at various wavelengths. This typically encompasses wave numbers ranging from 14,000–25 cm^−1^, and an area between 700 and 400,000 nm.

Infrared radiation (IR) is a form of energy or light that is invisible to the naked eye. The vibrational modes of the molecules (i.e. the stretching and bending of the molecule's electric dipole) determine the frequency of the IR absorbed by molecules. The ease with which energy is absorbed by the molecules determines the intensity of absorption. In turn, this is determined by the degree to which the molecule's dipole moment shifts during radiation absorption. FTIR, a widely used analytical spectroscopy technique, measures the energy of infrared light as it interacts with molecules. Afterwards, this vibration is employed to track catalytic activity and identify compounds in intricate mixtures [35]. Using FTIR spectra, the functional groups of the samples were examined in the present study, as the Mo-ion concentration in WO_3_ varied from 0 % to 20 %. The FTIR spectra of the Mo-doped and unadulterated WO_3_ films are shown in Fig. 2.

**Fig. 2:** FTIR spectra of WO_3_ thin film with different Mo-content.

As shown in the results, the band range that developed between 3296.76 and 3424.34 cm^−1^ is associated with surface hydroxyl group vibration, most likely as a result of water reabsorption from the surrounding atmosphere [36]. The deviation caused by an increase in Mo-ion concentration and the vibration of the tungsten hydroxyl bond (W-OH) is linked to the band that emerged in the range of 1558.62–1645.56 cm^−1^. The W-O-W bridge mode is also represented by a prominent band in the spectrum, which spans 850 to 650 cm^−1^ [37,38]. Only one peak is found for the presence of MoO_3_. Thus, the FTIR results verify that Mo has been substituted at the regular lattice site of WO_3_ and at the composition of WO_3_.

### 3.3 Effects of temperature and composition on dc-electrical conductivity

The electrical properties of Mo_x_W_1-x_O_3_ thin films were investigated using temperature-dependent resistivity. Fig. 3 presents how the absolute temperature affects these thin films' dark semi-logarithmic dc-electrical resistivity within the temperature range of 293–523 K. In particular, the magnitudes of the continuous electrical resistance of Mo_x_W_1-x_O_3_ thin films (0.0 % ≥ x ≥ 20 %) reveal an exponential behaviour that is very similar to that of ternary structure semiconductors. The linear part of the semi-logarithmic diagrams of dc-conductivity increase occurs as the temperature rises for all Mo_x_W_1-x_O_3_ samples, as can be clearly in Fig. 3A–E.

**Fig. 3:** The logarithmic scale of the dc-electrical resistivity of ternary MoxW1-xO3 thin films depends on absolute temperature. (A) x = 0.0, (B) x = 0.02, (C) x = 0.05, (D) x = 0.10 and (E) x = 0.20.

Furthermore, DC-electrical resistivity has a very similar behavior except for the magnitudes in the studied range for the Mo_x_W_1-x_O_3_ compositions (0 at.% ≥ x ≥ 20 at.%). As shown in Fig. 4 and Table 2, DC-resistivity decreases significantly with increasing temperature for each Mo-concentration ratio for all Mo_x_W_1-x_O_3_ samples. This finding indicates that conduction occurs through an active process, which also explains the semiconducting behaviour of the bulk amorphous structure. As reported by a previous study on the crystal structure of this compound, the size of the crystal and the degree of crystallinity decrease with increasing Mo concentration [12]. This finding confirms that the same conduction mechanisms are dominant in all ternary bulk glasses studied [[39], [40], [41]]. Moreover, the DC-electrical resistivity (ρ_dc_) decreases slowly with increasing temperature but at varying rates. This means that conduction occurs in this region through the variable range hopping of charge carriers in localised states near the Fermi level, which is predicted by Mott's variable range hopping model [6,[42], [43], [44]].

**Fig. 4:** Variability in the dc-electrical resistivity at various temperatures with the percentage of the Mo concentration.

**Table 2:** Effect of Mo content on dc-electrical resistivity value and standard deviation (sd) at different temperatures.

Mo-content	293K	350K	400K	450K	500K	523K
**X=0.00**	**(7.33 ± 0.39)x10**^**6**^	**(1.87 ± 0.32)x10**^**6**^	**(1.18 ± 0.29)x10**^**5**^	**(1.99 ± 0.23)x10**^**3**^	**(6.10 ± 0.25)x10**^**2**^	**(2.45 ± 0.28)x10**^**2**^
**X=0.02**	**(5.12 ± 0.39)x10**^**7**^	**(2.18 ± 0.32)x10**^**6**^	**(1.34 ± 0.29)x10**^**5**^	**(4.25 ± 0.23)x10**^**3**^	**(7.88 ± 0.25)x10**^**2**^	**(3.53 ± 0.28)x10**^**2**^
**X=0.05**	**(7.75 ± 0.39)x10**^**7**^	**(4.03 ± 0.32)x10**^**6**^	**(2.06 ± 0.29)x10**^**5**^	**(7.83 ± 0.23)x10**^**3**^	**(3.36 ± 0.25)x10**^**3**^	**(7.82 ± 0.28)x10**^**2**^
**X=0.10**	**(1.79 ± 0.39)x10**^**8**^	**(5.48 ± 0.32)x10**^**6**^	**(6.26 ± 0.29)x10**^**5**^	**(8.82 ± 0.23)x10**^**3**^	**(3.42 ± 0.25)x10**^**3**^	**(1.29 ± 0.28)x10**^**3**^
**X=0.20**	**(2.11 ± 0.39)x10**^**8**^	**(3.24 ± 0.32)x10**^**7**^	**(8.11 ± 0.29)x10**^**5**^	**(9.38 ± 0.23)x10**^**3**^	**(3.86 ± 0.25)x10**^**3**^	**(2.90 ± 0.28)x10**^**3**^

At higher temperatures, electrical resistivity decreases at a faster rate through the remaining temperature range, indicating that the conduction process is due to the thermally assisted tunneling of charge carriers in extended states. Furthermore, the relationship between DC-electrical resistivity and Mo concentration percentages at different temperatures is shown in Fig. 4. The results confirms that: resistivity at lower temperatures; that is T slowly increases when Mo-content increases. However, when the temperature increases; the slope of the curves gradually increases, until 523K, at which point the resistivity decreases in a dramatic way. This phenomenon can be attributed to decreasing the electrical resistivity at lower temperatures due to the intrinsic nature of the samples [45]. In this temperature region, the number of charge carriers due to intrinsic defects is in adequate, and the mobility of charge carriers is low. Thus, there may be too few charge carriers in conduction band to give rise to appreciable conduction. However, at higher temperatures, the decrease in resistivity is due to the thermal excitation of charge carriers from the grain boundaries of the neutral region of the grains [42,45]. The low mobility of charge carriers is easily compensated for by the creation of a large number of charge carriers. Thus, It can be concluded that, the conduction processes of all samples occur through more than one conduction mechanism [42,43].

### 3.4 Sheet resistance

Sheet resistance is a common indicator of the electrical resistance of thin films with a consistent thickness. This property shows the resistance of a square piece of thin material on opposite sides of the square and, can be used to compare the electrical characteristics of devices whose sizes vary greatly. Sheet resistance can also be used to assesses the resistivity of thin films throughout a square region and ascertain the degree of thickness uniformity and surface roughness. To compute the sheet resistance of thin coatings, it is assumed that the current flows through the plate's plane rather than in a perpendicularly manner. The term is also frequently used to describe materials created by doping semiconductors.

The resistivity of the thin-film material can be computed using the following formula (Eq. (2)), which multiplies the sheet resistance (**R**_**Sh**_) and the film thickness (t). [46];

(2) $$\rho_{DC}=R_{Sh}.t$$

Instead of using ohmic resistance or resistivity, we can use sheet resistance because it can be measured indirectly or directly using a two-point probe sensor. Fig. 5A–E depicts the semi-logarithmic property of the sheet resistance of Mo_x_W_1-x_O_3_ thin films as the concentration of Mo ions changes. As shown in the results, the change in the linear part of the sheet resistance behaviour due to temperature is an exponential and decreasing function with the change in the proportion of Mo^+2^. The sheet resistance of pure tungsten oxide is lowest at 425K, but with the addition of molybdenum, it reaches 350K. This finding suggests that the Mo ion causes a rapid drop in sheet resistance. Furthermore, the insertion of the Mo ions reduces sheet resistance due to an increase in crystallinity and a decrease in both the optical band gap energy and internal stresses in thin films.

**Fig. 5:** The logarithmic scale of sheet resistance versus temperature at different Mo-ions concentration, (A) x = 0.0, (B) x = 0.02, (C) x = 0.05, (D) x = 0.10 and (E) x = 0.20.

### 3.5 Mechanisms of conductivity and activation energies

The following is an expression of the hopping resistivity as a function of temperature in all ranges from 293 to 523 K for the samples prepared via deposition and after annealing using the Arrhenius equation [[47], [48], [49]]:

(3) $$\rho_{dc}=\rho_{o}\;\exp\left(\frac{\Delta E_{o}}{K_{B}T}\right)+\rho_{1}\;\exp\;\left(\frac{\Delta E_{1}}{K_{B}T}\right)$$

Both terms result from different conduction mechanisms. Here, the high-temperature region, 393–523K, is described by the first term, whilst the low-temperature region (293–393K), is described by the second term of Equation (3), and the main process is band conduction across enlarged states.

The pre-exponential factors (ρo) and (ρ1) in Equation (3) are heavily influenced by the composition, and their values assist in deciding the type of conduction mechanism [[50], [51], [52], [53]]. Moreover, the activation energies for the two conduction regions are denoted by ΔE_o_ and ΔE_1_, respectively; the Boltzmann constant is denoted by K_B_, and the absolute temperature is denoted by T. Taking the logarithm of both sides of Equation (3), we can convert it into two straight parts as follows;

(4) $$\mathrm{Ln}\;\rho_{dc}=\mathrm{Ln}\;\rho_{o}+\frac{\Delta E_{o}}{K_{B}}.\frac{1}{T}+\mathrm{Ln}\;\rho_{1}+\frac{\Delta E_{1}}{K_{B}}.\frac{1}{T}$$

The variation of ln(ρ) vs. (1000/T), according to Eq. (4), for Mo_x_W_1-x_O_3_ thin film samples under investigation is shown in Fig. 6A–E. This illustration demonstrates that the Arrhenius Equation (3) predicts the presence of two temperature regions for each of the as-deposited and annealed states. The activation energy for the two conduction zones can be determined by the slope of the established straight lines. The pre-exponential factors can also be obtained by intercepting the obtained straight lines with the ln(ρ)-axis and extrapolating them [10,11,54]. Table 3 lists the calculated pre-exponential factor values along with the two conductive regions’ respective activation energies for each of the samples before and after annealing with a changing Mo-ion ratio. It is obvious that the values of ρ_1_ in the low temperature region are about 10^2^-10^4^ times lower than the ρ_o_ of the high temperature region for the samples before and after annealing due to the lower mobility and density of the delocalised states [[55], [56], [57]]. This finding demonstrates that conduction occurs in the high temperature region through the hop-conduction mechanism via localised states. Tunneling through the vacant levels of the adjacent adjoining center is the cause of the resistivity in these areas.

**Fig. 6:** Plots of Ln ρ versus (1000/T) for as-deposited and after annealing of Mo_x_W_1-x_O_3_ thin films as a function of concentration of Mo-ions. (A) x = 0.0, (B) x = 0.02, (C) x = 0.05, (D) x = 0.10 and (E) x = 0.20.

**Table 3:** Pre-exponential factors, activation energy values and temperature transition for the two conduction regions, (1) the first region is the high temperature that extends from about 393 to 523K and (2) the second region is the low temperature that extends from 293 to 393K, as well as the values of change in as-deposited and post-annealed temperatures of Mo_x_W_1-x_O_3_ thin films.

Mo-ion content	As deposited					After annealing				
	Higher Temperature		Lower temperature		T_C_(K)	Higher Temperature		Lower temperature		T_C_(K)
	ρ_o_ (ῼ.cm)	ΔE_o_(eV)	ρ_1_ῼ.cm)	ΔE_1_(eV)		ρ_o_ (ῼ.cm)	ΔE_o_(eV)	ρ_1_(ῼ.cm)	ΔE_1_(eV)	
**0.00**	**4.03 ± 0.3x10**^**2**^	**0.783 ± 0.03**	**36.59 ± 0.04**	**1.12 ± 0.02**	**393 ± 5**	**181.27 ± 0.5**	**0.735 ± 0.05**	**27.11 ± 0.3**	**0.935 ± 0.03**	**373 ± 5**
**0.02**	**7.35 ± 0.3x10**^**2**^	**0.761 ± 0.03**	**43.67 ± 0.04**	**1.09 ± 0.02**	**385 ± 5**	**221.41 ± 0.5**	**0.722 ± 0.05**	**29.96 ± 0.3**	**0.917 ± 0.03**	**368 ± 5**
**0.05**	**8.98 ± 0.3x10**^**2**^	**0.646 ± 0.03**	**54.59 ± 0.04**	**1.04 ± 0.02**	**373 ± 5**	**735.09 ± 0.5**	**0.663 ± 0.05**	**33.12 ± 0.3**	**0.913 ± 0.03**	**357 ± 5**
**0.10**	**9.89 ± 0.3x10**^**3**^	**0.509 ± 0.03**	**65.58 ± 0.04**	**0.92 ± 0.02**	**365 ± 5**	**1.09 ± 0.5x10**^**3**^	**0.575 ± 0.05**	**36.59 ± 0.3**	**0.909 ± 0.03**	**350 ± 5**
**0.20**	**5.98 ± 0.3x10**^**4**^	**0.281 ± 0.03**	**81.45 ± 0.04**	**0.85 ± 0.02**	**355 ± 5**	**3.64 ± 0.5x10**^**3**^	**0.530 ± 0.05**	**44.70 ± 0.3**	**0.847 ± 0.03**	**344 ± 5**

In Table 3, we note that the activation energy ΔE_1_ (at the lower temperature region) is slightly larger than ΔE_o_ (high temperature region) for the as-deposited and annealed states. They also decrease gradually with Mo-ion concentration. The decrease in the two activation energies is due to the increase in the Mo-ions resulting in a change in the stoichiometric property of the formed phase. Moreover, the values of the pre-exponential factors and activation energy after thermal annealing are lower than in the as-deposited state in the whole temperature range. This result is due to the improvement in the degree compound of crystallinity, the increase in crystalline agglomerations, crystallite size and optical band gap energy and a decrease in internal stresses and the treatment of crystalline defects. However, as a function of Mo-ion concentration, the conductivity mechanism's transition temperature (Tc) changes, as seen in Fig. 6 and Table 3.

From Fig. 7, the measured data of the as deposited and annealed sample were fitted to obtain straight lines, thus satisfying from Equations. (5), (6)). [58,59];

(5) T_C_ = 387.55–180.46. X (As deposited)

(6) T_C_ = 368.83–140.98.X (After annealing)

**Fig. 7:** The transition temperature of conductivity mechanisms versus Mo ions concentration of as deposited and after annealing.

These findings can be explained as follows: because the size of the Mo and W atoms is equal, the Mo atom is implanted within the host unit cell of WO_3_ rather than the W atom. Thus, with the same extension, the unit cell's dimensions remain the same in all three directions. As a result, a rise in the doping percentage which in the composite phase represents impurities and non-stoichiometry and causes the shift in the transition temperature, Tc. Thus, given that the temperature, contaminants, and crystal defects all affect the conductivity mechanism, the change in impurity content that influences the conductivity mechanism can be linked to the shift in Tc.

### 3*.6. Hopping conduction* via *localised states*

3.6

This technique can be found in the higher temperature range (393–523K), as described in the first term of Equation (3). It progresses via hopping conduction localised states, and the inherent temperature is reached after the impurity exhaustion temperature [60]. When the amount of Mo in WO_3_ increases from zero to 20 %, the activation energy ΔE_o_ values for the as-deposited sample decreases from 0.783 to 0.283eV, whilst the pre-exponential parameter, ρ_o_ for the as-deposited sample increases from 4.03 × 10^2^ to 5.98 × 10^4^ (Ω cm) in this region. The increase in atomic bonding disorder between neighbours and a variety of complex stoichiometries may be responsible for the lower activation energy values. In turn, these increase the density of neighboring tail states and establish a linear relationship between the two values and the Mo content in the WO_3_ matrix. Similarly, after thermal annealing, the values of *ΔE*_*o*_ decrease from 0.735 to 0.530 eV, whereas the pre-exponential factor increases from 1.81 × 10^2^ to 3.64 × 10^3^ (ῼ.cm) with the increase in Mo-ion concentration. These results align well with those reported in earlier research [6,[61], [62], [63]].

Fig. 8A–D also shows the changes in the pre-exponential factors, (ρ_o_) and activation energy (ΔE_o_) values in high-temperature regions with Mo content for the as-deposited and annealed Mo_x_W_1-x_O_3_ thin films. Fitting was done for the results, and the increase in the exponential factor was linear. We also found empirical equations describing the variation in Mo content in these figures. Similarly, fittings were made for the results of the two estimated activation energies, and experimental equations were written in the figure showing the linear decrease with the increase in the percentage of Mo-ions. In the empirical equations, X denotes the percentage of Mo content in the Mo_x_W_1-x_O_3_ thin films. These results are consistent with earlier research [55,64].

**Fig. 8:** At higher temperature region; plot the changes of pre-exponential factors, ρ_o_ and activation energies, ΔE_o_ for as-deposited (B, D) and after annealing (A, C) as a function of Mo-ions concentration.

### 3.7 Hopping conduction near the Fermi level

The second term of Equation (3) provides the dc-resistivity for the lower temperature range between 393K and room temperature (293K). The conduction mechanism in this instance extends upward to the impurity exhaustion temperatures and is comparable to impurity conduction in semiconductors that have been heavily doped. Due to the ionisation of impurity atoms, this region is known to have a semiconductor's extrinsic conductivity. In the current study, the results indicate that the obtained values ΔE_1_ for the as-deposited sample decrease from 1.12 to 0.85 eV, whilst the pre-exponential factor's (ρ_1_) values increase from 36.59 to 81.45 (Ω cm). In addition, the value of ΔE_1_ after annealing is reduced from 0.94 to 0.85 eV, whilst the values of the pre-exponential factor (ρ_1_) increase from 27.11 to 44.70 (Ω cm) with the increase in the percentage of Mo-ion. Another important observation from Table 2 is that, in line with Mott's prediction, the pre-exponential factor is smaller in the lower temperature range (below 393 K) than in the higher temperature range, in the order of 10^2^, both before and after annealing [6,65,66]. Additionally, the energy of activation values of the current Mo_x_W_1-x_O_3_ thin films are lower than those in the high-temperature region, (i.e. above 393K). This finding illustrates how variable range hopping, thermionic emission and conduction mechanisms operate at different temperatures as thermally activated processes [64,67]. The obtained activation energy values further demonstrate that semiconductors are present in the produced samples.

Fig. 9A–D further displays how the values of ρ_1_ and ΔE_1_ vary for both the as-deposited and annealed samples in the low temperature region (from 293 to 393K) with Mo content for Mo_x_W_1-x_O_3_ thin films. The value of the pre-exponential factor increases as a linear relationship, whilst the value of the activation energy also decreases linearly with the concentration of the Mo-ion. By fitting the results and writing experimental equations, we can describe the variation of the relationship within the shapes with the change in Mo-ion content. In the experimental equations, X is an indicator of the Mo-content percentage in the Mo_x_W_1-x_O_3_ thin films. Due to an increase in collisions between charge carriers and vibrating atoms brought on by thermal heating as well as an increase in the concentration of impurity atoms, the residual electrical resistivity of the as-deposited or annealed samples increases. As temperatures rise, the degree of crystallization improves and the number of crystallite clusters increases, resulting in a decrease in the activation energy needed for an electron. These results are in line with those reported in earlier research [39,[68], [69], [70]].

**Fig. 9:** At lower temperature region; Plot the variation of pre-exponential factors and activation energies for as-deposited (B, D) and after annealing (A, C) as a function of Mo-ions concentration.

### *3.8* Determining the Mott's parameters

The stoichiometry of the metals and oxygen, as well as any purity that may be present in the input materials, can directly influences the physicochemical characteristics of the thin films transition metal oxides'. Chemical impurities start to show up in thin films when stoichiometry is absent. Furthermore, the preparation conditions cause crystalline defects to form, which have an impact on the development of the thin film matrix (the amorphous and crystalline mixtures). The position of the Fermi level is also altered by the presence of amorphous Mo_x_W_1-x_O_3_ atoms. Thus, electrons may be redistributed to localised states as a result of the dispersion of structural defects in thin films created during the growth process. During this process, the electrical properties of thin films are significantly influenced by structural flaws. Based on Matthiessen's rule, impurities, crystal defects, temperature, and phonons (lattice vibrations) are just a few of the variables that can affect the electrical conductivity, (σ), of semiconductor materials [41,43]. At lower temperatures, the only factors affecting electrical conductivity are impurities and structural flaws.

In addition, there might not be many charge carriers in the conduction band, which allows impurities to play a role in the electrical conductivity mechanism. Therefore, below 335 K, jumping charge carriers are responsible for the resulting current passing through the thin films. These use phonons to help them transition between impurities because they lack the energy necessary to induce the excitation of the adjacent band. At the same time, the temperature rises, conductivity increases quickly. Thus, is easy to compensate for the low mobility of charge carriers by producing a large number of them. The specimen's conductivity increased also as a result [[71], [72], [73]]. The electrical conductivity of as-deposited and annealed Mo_x_W_1-x_O_3_ thin films through two different temperature regions, (the low-temperature region starts from 293 to 393K, whilst, the high temperature region starts from 393 to 523K), may be thoroughly explained by Mott's model. Based on Mott's theorem, the electrical conductivity σ is given by Eqs. (7), (8)) [74,75].

(7) $$\sigma T^{1/2}=A.\exp\left[-{\left(\frac{T_{o}}{T}\right)}^{1/4}\right]\text{;}$$

(8) $$\mathrm{Ln}\;\sigma T^{1/2}=\mathrm{Ln}\;A-T_{o}^{\frac{1}{4}}.T^{-1/4}$$

where T_o_ is a characteristic temperature that indicates the sample's level of disorder, and A is a constant connected to the Fermi level localised state density. The relationship between (T_o_) and (A) is given by Eqs. (9), (10)) [6,75,76].:

(9) $$A=3e^{2}\nu_{o}\sqrt{\frac{N\left(E_{F}\right)}{8\pi \alpha TK_{B}}}\;{\left(\Omega .cm\right)}^{-1}.K^{1/2}$$

(10) $$T_{o}=\frac{m\alpha^{3}}{K_{B}N\left(E_{F}\right)}\;\left(K\right)$$

where e is the electronic charge, N(E_F_) is the localised state density at the Fermi level, which is estimated by adjusting the parameter electronic wave decay length α^−1^ for localised states; ν_o_ is the typical phonon frequency called Debye frequency (ν_o_ ~ 10^13^ Hz); m is the dimensionless constant in the range of 2.06–4.2 depending on the N(E_F_) feature. , α is the decay constant of the wave function of localised states near the Fermi level (0.3 nm ≤ α^−1^ ≤ 3 nm) [70]; and K_B_ is the Boltzmann constant [6,75,76]. Solving Equations (9), (10) simultaneously, to obtained the following; $\alpha =709.56.\;A.\;T_{o}^{\frac{1}{2}}\left({cm}^{-1}\right)$ and $N\left(E_{F}\right)=9.089x10^{16}A^{3}T_{o}^{1/2}\;\left({eV}^{-1}{cm}^{-3}\right)$. The average hopping distance (R) relies on the density and distribution of states and is given by Eq. (11):

(11) $$R=\sqrt[{4}]{\frac{9}{8\pi \alpha K_{B}N\left(E_{F}\right)}}\;\left(cm\right)\text{.}$$

The hopping energy W can be computed using the value of N(E_F_) (cm^−3^eV^−1^), which is given as Eq. (12):

(12) $$w=\frac{3}{4\pi R^{3}N\left(E_{F}\right)}\;\left(eV\right)\text{.}$$

The kind of conduction mechanism can be established by plotting ($\mathrm{Ln}\;\sigma T^{1/2}$) vs. $T^{-1/4}$ for the present thin film sample. The electrical conductivity of Mo_x_W_1-x_O_3_ and the temperature dependence of thin films are clearly positive and exhibit unusual metallic conduction characteristics. At the same time, the values of T_o_ and A can be estimated from the slope of a linear fit of the straight lines and a portion of their intercept to the y-axis of the plots shown in Fig. 10A–E and listed in Table 4.

**Fig. 10:** Plots of Ln σT^1/2^ vs T^−1/4^ for as-deposited and after annealing of Mo_x_W_1-x_O_3_ thin films at different Mo-concentration: (A) x = 0.00, (B) x = 0.02, (c) x = 0.05, (D) x = 0.10 and (E) x = 0.20.

**Table 4:** Mott's parameters such as localized states density near the Fermi level N(E_F_), residual conductivity, A(ῼ.cm)^−1^, characteristic temperature, T_o_(K), degree of localization, α (cm^−1^), hopping energy, W(meV), average hopping distance, R(cm) and αR estimated for as-deposited and after annealing temperature of Mo_x_W_1-x_O_3_ thin films.

Mo-ion	N(E_F_)x10^13^ (eV cm)		Ax10^−3^ (ῼ.cm)^−1^		T_o_x10^10^ (K)		αx10^5^ (cm^−1^)		W (meV)		Rx10^−5^ (cm)		αR	
	As	Ann	As	Ann	As	Ann	As	Ann	As	Ann	As	Ann	As	Ann
**0.00**	**433.9 ± 2**	**14.19 ± 0.5**	**246.6 ± 2**	**110.8 ± 3**	**5.90 ± 2**	**2.54 ± 3**	**10.02 ± 0.4**	**2.42 ± 0.3**	**1.80 ± 0.2**	**1.46 ± 0.2**	**3.13 ± 0.5**	**10.49 ± 2**	**31.33 ± 2**	**25.39 ± 2**
**0.02**	**271.2 ± 2**	**6.34 ± 0.5**	**0.18 ± 2**	**0.110 ± 3**	**5.66 ± 2**	**2.29 ± 3**	**8.45 ± 0.4**	**1.79 ± 0.3**	**1.78 ± 0.2**	**1.42 ± 0.2**	**3.67 ± 0.5**	**13.84 ± 2**	**31.02 ± 2**	**24.73 ± 2**
**0.05**	**43.24 ± 2**	**1.32 ± 0.5**	**0.027 ± 2**	**0.015 ± 3**	**2.90 ± 2**	**2.00 ± 3**	**3.67 ± 0.4**	**1.01 ± 0.3**	**1.51 ± 0.2**	**1.37 ± 0.2**	**7.16 ± 0.5**	**23.60 ± 2**	**26.23 ± 2**	**23.91 ± 2**
**0.10**	**29.18 ± 2**	**0.38 ± 0.5**	**0.030 ± 2**	**0.064 ± 3**	**2.40 ± 2**	**1.78 ± 3**	**3.02 ± 0.4**	**0.64 ± 0.3**	**1.44 ± 0.2**	**1.33 ± 0.2**	**8.29 ± 0.5**	**36.24 ± 2**	**25.04 ± 2**	**23.23 ± 2**
**0.20**	**7.165 ± 2**	**0.29 ± 0.5**	**0.061 ± 2**	**0.068 ± 3**	**1.60 ± 2**	**1.22 ± 3**	**1.65 ± 0.4**	**0.49 ± 0.3**	**1.30 ± 0.2**	**1.21 ± 0.2**	**13.69 ± 0.5**	**42.97 ± 2**	**22.60 ± 2**	**21.14 ± 2**

Table 4 shows that the residual conductivity (A) values and the characteristic temperature (T_o_) in the two temperature regions decrease with the concentration of Mo-ions. The limitations placed on the thermal vibration of metal ions, which have an adverse effect on the motion of free electrons, are responsible for such behaviour. Based on the delocalised electrons, there is no insulator-metal transition, transition metal oxides often have relatively poor conductivities, and disorder grains enhance the confusion of passing currents, thus increasing resistance. The results obtained are in good agreement with those of other investigators [6,[76], [77], [78], [79]]. A cursory review of the data shown in Table 4 shows that when the Mo-percentage increases, all predicted parameters, except for the hopping distance (R) decrease. Mott's variable range hopping conduction model states that the values of the hopping energy (W) and the product (αR) must be larger than (K_B_T) and unity, respectively. Thus, the changeable range of hopping conduction is the cause of the conduction mechanism [6,[80], [81], [82], [83], [84]]. Given that W > K_B_T and αR>1 is satisfied, it can be concluded from Table 4 that the current results for all Mo_x_W_1-x_O_3_ thin film samples agree well with the VRHC model proposed by Mott [6,80,81,83,85].

The localised density of states N(E_F_) decreased from 4.339 × 10^15^ to 7.165 × 10^13^ (eV^−1^ cm^−3^) and from 14.188 × 10^13^ to 2.48 × 10^12^ (eV^−1^ cm^−3^) as the Mo content increased, respectively. These findings are similar to those reported in other studies [64,68,69]. Thus, the conduction mechanism is brought on by the variable range hopping conduction of Mo_x_W_1-x_O_3_ thin films [44,[81], [82], [83]].

Fig. 11 demonstrates the relationship between the average hopping energy (W) and the disorder degree parameter (T_o_) in relation to the Mo-content percentage in the Mo_x_W_1-x_O_3_ thin film samples. This chart demonstrates the linear relationships between (To) and the Mo-content percentage and (W) and Mo-percent. Equations (13), (14)) are the empirical equations that characterize the linear connections that best suit the given data:

(13) $$T_{o}=5.282x10^{10}-2.15x10^{11}\;X\;\left(K\right)\;\left(As\;deposited\right)$$

(14) $$T_{o}=2.428x10^{10}-6.24x10^{10}\;X\;\left(K\right)\;\left(After\;annealing\right)$$

where X = 0.0, 0.02, 0.05, 0.10 and 0.20, referring to the percentage of Mo-content within the Mo_x_W_1-x_O_3_ thin films.

**Fig. 11:** The characteristic temperature of as deposited and after annealing as a function of Mo-concentration.

### 3.9 Trapping states and potential barrier energies

One possible explanation for the steady increase in Dc conductivity along with temperature is the effect of carrier trapping in grain boundaries, which results from their capture at the trapping states found at the grain borders, thus depopulating the area inhabited by the charge carriers. The grain effect disappears completely as the number of trapped charge carriers (N) increases and approaches the critical point. As the concentration of trapped charge carriers (N) increases to the critical concentration of acceptors or donors (N*), the grain is said to have lost all of its population. In this instance, the acceptor or donor concentration (N*) and the Dc-electrical conductivity, or σ, at the grain boundaries can be determined using Eq. (15) [84,85].:

(15) $$\frac{\sigma }{T}=A\;\exp\;\left[\frac{\left(-\frac{E_{g}}{2}+e_{T}\right)}{K_{B}T}\right]$$

where T is the absolute temperature, E_g_ the band gap energy, A is a new pre-exponential factor, e_T_ the trapping state energy in the grain boundary, and K_B_ is the Boltzmann constant.

Fig. 12A–E, presents an illustration of ln(σ/T) vs the lower temperature's reciprocal of the absolute temperature (1000/T) (ranging from 293 to 393K). This figure displays a straight line with a slope of [(−E_g_/2) + e_T_]/K_B_ and intercepts the ln(σ/T)-axis in a value equals ln(A). Therefore, the trapping state energies (e_T_) can be calculated for Mo_x_W_1-x_O_3_ thin films using the optical band gap energies slope (Eg) as a guide [24,86]. The determined values of the trapping state energies(e_T_) and the pre-exponential factor (A) are shown in Table 5.

**Fig. 12:** The representation of Ln (σT) versus (1000/T) for as deposited and after annealing Mo_x_W_1-x_O_3_ thin films. (A) x = 0.00, (B) x = 0.02, (c) x = 0.05, (D) x = 0.10 and (E) x = 0.20.

**Table 5:** The pre-exponential factor and the trapping state energy for as deposited and after annealing of Mo_x_W_1-x_O_3_ thin films.

Mo-ion	Eg (eV) (Ref 7)	Exponential factor; A(Ω·cm·K)^−1^		Trapping state energy e_T_(eV)		Pre-exponential constant; B (Ω·cm)^−1^ K^−1/2^		Potential barrier energy; eϕ_B_ (eV)	
		As	Ann	As	Ann	As	Ann	As	Ann
**0.00**	**2.76 ± 0.03**	**4.41 ± 1.8x10**^**2**^	**16.97 ± 3**	**2.38 ± 0.05**	**2.22 ± 0.03**	**15.29±2x10**^**3**^	**5.88±2x10**^**2**^	**0.82 ± 0.02**	**0.74 ± 0.02**
**0.02**	**2.66 ± 0.03**	**16.06 ± 1.8x10**^**2**^	**181.93 ± 3**	**2.30 ± 0.05**	**2.16 ± 0.03**	**42.44±2x10**^**3**^	**7.44±2x10**^**2**^	**0.89 ± 0.02**	**0.83 ± 0.02**
**0.05**	**2.64 ± 0.03**	**22.58 ± 1.8x10**^**2**^	**306.82 ± 3**	**2.22 ± 0.05**	**2.13 ± 0.03**	**55.69±2x10**^**3**^	**6.31±2x10**^**3**^	**0.90 ± 0.02**	**0.84 ± 0.02**
**0.10**	**2.58 ± 0.03**	**42.44 ± 1.8x10**^**3**^	**426.78 ± 3**	**2.19 ± 0.05**	**2.10 ± 0.03**	**78.31±2x10**^**3**^	**8.05±2x10**^**3**^	**0.99 ± 0.02**	**0.85 ± 0.02**
**0.20**	**2.56 ± 0.03**	**80.18 ± 1.8x10**^**3**^	**744.36 ± 3**	**2.08 ± 0.05**	**1.99 ± 0.03**	**27.81±2x10**^**5**^	**11.35±2x10**^**3**^	**1.03 ± 0.02**	**0.86 ± 0.02**

Fig. 13A and B displays how the pre-exponential factor (A) changes in relation to the Mo-content percentage for the as-deposited and after annealed samples. Fig. 13A and Table 5 show that, the increase in the exponential factor (A) is in the order of 10^4^ and 10^2^ in the as-deposited and in annealed samples upon increasing the Mo content. When X is raised from 0 % to 20 %, the pre-exponential factor (A) increases from 4.41 × 10^2^ to 80.18 × 10^3^ (Ω cm K)^−1^ for the as deposited sample and from 16.97 to 744.36 (Ω cm K)^−1^ for the annealed sample.

**Fig. 13:** The variation of pre-exponential factor for as deposited, (A), and after annealing, (B), as a function of Mo-concentration of Mo_x_W_1-x_O_3_ thin films.

In addition, Fig. 14 A and B shows how the energy of the trapping state varies with the Mo content percentage. Equations (16), (17)) explains the observed practically linear decrease in trapping state energy as the Mo-content percentage increases:

(16) $$e_{T}=2.333-1.356\;X\;\left(eV\right)\;\left(As\;deposited\right)$$

(17) $$e_{T}=2.194-0.993\;X\;\left(eV\right)\;\left(After\;annealing\right)$$

where X is the Mo content percentage that provided in WO_3_. From Equation (18), the values of the trapping state energies of WO_3_ and MoWO_3_ can be theoretically estimated. For MoWO_3_ as deposited sample, put X = 0, so e_T_ = 2.333eV, whilst for the MoWO_3_ X = 0.20, so e_T_ = 2.0618eV. In comparison, after annealing at X = 0, so e_T_ = 2.194eV and for X = 0.2, e_T_ = 1.9954eV. The decreasing dc-conductivity is confirmed by the decreasing value of the trapping state energy when increasing the Mo content in the MoWO_3_ thin films. The phenomenon of charge carrier trapping in grain boundaries can be attributed to this behaviour, because it results in a depopulated area of these carriers, as they are captured at the traps located at the grain boundaries [74,84]. However, when the grains are largely depopulated (N > N*), the electrical conductivity at the grain borders follows Seto's formula [85].:

(18) $$\sigma .T^{1/2}=B\;\exp\left[\frac{-e\Phi_{B}}{K_{B}T}\right]$$

where (eΦ_B_) is the energy of the potential barrier, T is the absolute temperature, and another pre-exponential constant, (B), is dependent on the electrical conductivity of the materials under investigation's.

**Fig. 14:** The variation of trapping state energy for as deposited, (A), and after annealing, (B), of Mo_x_W_1-x_O_3_ thin films.

Fig. 15A–E presents the linear relationship between ln (σ.T^0.5^) and the reciprocal of the absolute temperature (1000/T) of the Mo_x_W_1-x_O_3_ thin films samples. The concept of partially depopulated grains is the foundation for DC-electrical conductivity. As can be seen, within the current temperature range under study (293K–393K), this provides a strong correlation with the observed experimental results. The slope of the straight lines produced in Fig. 16 is employed to calculate the grain boundary's potential barrier energy (eφ_B_). Table 5 presents the resulting values.

**Fig. 15:** Plots the relation Ln(σ.T^1/2^) versus (1000/T) according to Seto's formula as a function Mo-ions concentration. (A) x = 0.00, (B) x = 0.02, (c) x = 0.05, (D) x = 0.10 and (E) x = 0.20.

**Fig. 16:** The variation of pre-exponential constant, versus the Mo-ions concentration for as deposition, (A), and after annealing, (B).

Fig. 16Aand B shows the changes in the potential energy barrier (eϕ_B_) and the pre-exponential constant (B) in terms of the Mo-content percentage in the MoxW_1-x_O_3_ thin films sheets. Based on the following empirical equations (19), (20)), straight lines are obtained by fitting the variation of (B) and (eϕ_B_) as shown below:

(19) $$B=\left(4.14x10^{5}+1.36.X\right){\left(\Omega .cm\right)}^{-1}.K^{-\frac{1}{2}}\;\left(As\;deposited\right)$$

(20) $$B=\left(1.34x10^{3}+5.50x10^{4}X\right){\left(\Omega .cm\right)}^{-1}.K^{-\frac{1}{2}}\;\left(After\;annealing\right)$$

where X = 0,0.02,0.05,0.1 and 0.2 at.% which is the proportion of the Mo-content in the WO_3_ thin films. When X = 0, for WO_3_ one can get B = 4.14 × 10^5^ (Ω cm)^−1^ K^−1/2^ for as deposited sample and B = 1.34 × 10^3^ (Ω cm)^−1^ K^−1/2^ for the annealed sample. In addition, when x = 0.2, B = 4.14 × 10^5^ (Ω cm)^−1^ K^−1/2^ for the as deposited sample and B = 12.34 × 10^3^(Ω·cm)^−1^ K^−1/2^ for annealed Mo_x_W_1-x_O_3_ thin films samples.

The variation of potential barriers, eϕ_B_ as a function of Mo-ions concentration for the as deposited and annealed of Mo_x_W_1-x_O_3_ thin films can be seen in Fig. 17A and B.

**Fig. 17:** The variation of potential barrier energy (Φ_B_) versus the Mo-content for the as deposited, (A), and after annealing, (B), of Mo_x_W_1-x_O_3_ thin films.

By fitting the relation, we have the following empirical equations (21), (22)):

(21) $$e\phi_{B}=0.853+1.006.X)\left(eV\right)\;\left(As\;deposited\right)$$

(22) $$e\phi_{B}=0.792+0.353.X)\left(eV\right)\;\left(After\;annealing\right)$$

where x is the concentration of Mo-ions. At x = 0.0, the potential barrier energies are 0.853 eV and 0.792eV for as deposited and annealed WO_3_ thin films, respectively. In comparison, at x = 0.2, the potential barriers are 1.0542 and 0.8626eV for the annealed process. When the Mo-ratio grew, so did the potential barrier energy (eΦ_B_). These outcomes match other semiconducting systems well and are consistent with the findings of past works [[85], [86], [87]].

## 5 Conclusion

This study investigated the preparation of thin films from Mo_x_W_1-x_O_3_ (0 ≥ x ≥ 20 at. %) using spray pyrolysis and a 2-h thermal annealing process at 823 K. The study's conclusions are as follows.

(1) FTIR analysis results: The vibration of the surface hydroxyl group ranges from 3296.76 to 3424.34 cm−1, whilst the vibration of the tungsten hydroxyl bond (W-OH) ranges from 1558.62 to 1645.56 cm−1. In addition, the W-O-W bridge mode is represented by a prominent band in the spectrum, extending from 850 to 650 cm^−1^. Furthermore, no peak appeared to indicate the presence of MoO_3_ thin films.
(2) The surface morphology study of pure and doped WO_3_ using FE-SEM shows island-like structure of minute microparticles, which depends on the effects of incorporation of Mo ions into the WO_3_ samples. But when 20 % molybdenum is added, the film takes the form of a dense network of islands with nest-like roots. Thus, the improved cross-channeling of the 20 % Mo-doped film provides broad paths for ions to easily diffuse into the film network along with accelerated kinetics that improves the electrical performance of the thin films.
(3) – Based on analysis of the proportions of element components via EDX, the proportions of the discovered elements (Mo, W, and O) and the elements selected through the experiment showed good agreement. The results also unequivocally showed that the 20 % Mo sample and the uncoated sample are single-phase samples that are free of additional elemental contaminants. In addition, the oxygen percentages are marginally larger than the atomic percentages
(4) - The electrical conductivity mechanisms of Mo_x_W_1-x_O_3_ thin films are divided into two categories: low-temperature mechanisms, which start from 293 to 393K, and high-temperature mechanisms, which start from 393 to 523K. As more Mo ions are added, DC electrical conductivity decreases, along with the decrease in pre-exponential factors (σ_o_ and σ_1_) and activation energies (ΔE_o_ and ΔE_1_). Analysis of the DC electrical conductivity data of the Mo_x_W_1-x_O_3_ thin film in the temperature range of 293K–523K indicates that both temperature and Mo content have a significant influence on the electrical conduction mechanism. This is because the variable mobility of local states serves as the main conduction mechanism at low temperatures. At high temperatures it causes the transition temperature to drop to 344K due to localized states from the impurity depletion temperature to the intrinsic temperature, which occurs when conduction stops.
(5) - Mott's model has been effectively applied to the electrical data for this region. The barrier potential, trapping state energy, and Mott parameters are calculated and discussed. The results show that increasing the percentage of Mo content increases the potential barrier energy (eϕ_B_) and average hopping distance (R), while simultaneously reducing the degree of disorder parameter (T_o_), the energy of trapping states (e_T_), and the degree of localization (α^−1^), Furthermore, we identified the product of the average mobility energy (W) (αR), which confirms that the Mott's variable hopping conduction is followed by the current samples.
(6) - All the parameters studied for n-type thin-film semiconductors in this work are highly recommended for use in various optical applications, such as thin-film solar cells used as window layer.

## Data availability

Data will be made available on request.

## CRediT authorship contribution statement

**S.M. Alshomar:** Visualization, Validation, Methodology, Funding acquisition, Alaa Ahmed Akl, Writing – review & editing, Resources, Funding acquisition. **Mohamed S. Attia:** Investigation, Formal analysis, Conceptualization. **Naglaa Fathy:** Visualization, Supervision, Resources. **Hissah Saedoon Albaqawi:** Methodology, Formal analysis, Conceptualization. **Hira Affan:** Validation, Resources, Methodology. **Ehab Sabry Mohamed:** Writing – review & editing, Writing – original draft. **Lamiaa G. Amin:** Writing – review & editing, Writing – original draft, Visualization, Investigation. **Safwat A. Mahmoud:** Writing – review & editing, Writing – original draft, Resources, Project administration, Data curation, Conceptualization.

## Declaration of competing interest

The authors declare that they have no known competing financial interests or personal relationships that could have appeared to influence the work reported in this paper.
